# Exploration for Countering the Episodic Memory

**DOI:** 10.1155/2022/7286186

**Published:** 2022-03-24

**Authors:** Rong Zhou, Yuan Wang, Xiwen Zhang, Chao Wang

**Affiliations:** ^1^Mechanical Engineering School, Southeast University, Nanjing, China; ^2^Aviation Engineering School, Air Force Engineering University, Xi'an, China; ^3^Information and Navigation College, Air Force Engineering University, Xi'an, China

## Abstract

Reinforcement learning is a prominent computational approach for goal-directed learning and decision making, and exploration plays an important role in improving the agent's performance in reinforcement learning. In low-dimensional Markov decision processes, table reinforcement learning incorporated within count-based exploration works well for states of the Markov decision processes that can be easily exhausted. It is generally accepted that count-based exploration strategies turn inefficient when applied to high-dimensional Markov decision processes (generally high-dimensional state spaces, continuous action spaces, or both) since most states occur only once in deep reinforcement learning. Exploration methods widely applied in deep reinforcement learning rely on heuristic intrinsic motivation to explore unseen states or unreached parts of one state. The episodic memory module simulates the performance of hippocampus in human brain. This is exactly the memory of past experience. It seems logical to use episodic memory to count the situations encountered. Therefore, we use the contextual memory module to remember the states that the agent has encountered, as a count of states, and the purpose of exploration is to reduce the probability of encountering these states again. The purpose of exploration is to counter the episodic memory. In this article, we try to take advantage of the episodic memory module to estimate the number of states experienced, so as to counter the episodic memory. We conducted experiments on the OpenAI platform and found that counting accuracy of state is higher than that of the CTS model. At the same time, this method is used in high-dimensional object detection and tracking, also achieving good results.

## 1. Introduction

Reinforcement learning, widely used in terms of the optimal control of Markov decision processes (MDPs) such as games and robotics, is a prominent computational approach for goal-directed learning and decision making [1].

The agent in reinforcement learning interacts with an environment, rather than just accepts a supervised signal, learning to map situations of a trajectory (or for some situations an episode) to actions to achieve a maximum expected cumulative reward.

When meeting high-dimensional situations, approximate solution methods were required. Deep Q-network (DQN) [2, 3] first attempted to apply reinforcement learning to high-dimensional problems by combining Q-learning with deep convolutional neural networks (CNN) as parameterized function approximators. However, this gives rise to more uncertainty of the reinforcement learning process.

All the time, in both low and high dimensions, tradeoff between exploration and exploitation is a great challenge arising in reinforcement learning for the agents interacting with unknown environments [1].

Hyperopic exploration, a main challenge in reinforcement learning, is essential for the extensively used gradient based reinforcement learning algorithms being sensitive to the initial policy, flat or deceptive gradient, and also for the uncertainty of action values estimation, to make sure that the agent is not trapped into local optimization.

In terms of the difficulty of exploration, [4] roughly classified Atari 2600 games in Arcade Learning Environment (ALE) into three taxa: easy exploration (this taxon can be divided into two according to the final scores), hard exploration with dense reward, and hard exploration with sparse reward. It is obvious that, for the above traps, different exploration strategies work. Just few strategies such as pseudocount-based exploration [4] are valid for the well-known hard exploration Montezuma's Revenge, while most strategies can surpass human optimum in easy exploration game Pong. Environments such as robotics and real scenarios can be more complex than Atari. The reinforcement learning environment is commonly equipped with sparse reward, deceptive reward, confused state, complex state distribution, etc.; all these traps may bring oscillatory output or local optimum; however, most existing exploration methods just concentrate on one trap. We will focus on the combination of them in this article.

Existing tremendous exploration methods are spontaneously divided into two categories: endogenous exploration and exogenous exploration, in terms of the generation of exploration's action derived from intrinsic factors of the environment or not, such as states and goals.

Representative endogenous exploration focuses on the guidance “explore what surprises you” [1], such as curiosity-driven/intrinsic motivation/novelty-based methods [5–13].

State-based intrinsic exploration strategies use various indicators such as prediction error and information gain to describe the intrinsic reward signal. Exploration based on the variation in agent prediction error or learning progress is a typical method.

Following the strong representation ability of neural networks, state-of-the-art literature focuses on learning the intrinsic reward/exploration bonus from the state/state-action pairs, rather than applying the predefined indicators. References [5, 9] experiment on ignoring the extrinsic reward to keep away from getting stuck in the deceptive reward problems.

For most of the “real scenarios,” this hypothesis is reasonable, and the intrinsic reward motivated by the final goal is actual existence; that is to say, the goal of the learning phase is observable. The computed intrinsic reward may not encourage the agent to explore in a high-return direction. However, for the environments whose goals/high reward states cannot be observed or inferred from state, these curiosity-driven methods may be powerless. A typical example in OpenAI Gym [14] is the benchmark Mountain Car environment; its states are continuous and actions are discrete. This game guides an underpowered car to reach goal on the top of a mountain. Horizontal position and velocity compose the state space, and their values are continuous. Legal actions are {−1, 0, 1} which represent a scalar acceleration. The agent may be trapped into local optimization if the car does not reach the mountaintop goal as quickly as possible.

State of this environment has no indistinctive features to depict a goal, although the rendered frame shows a red flag to the programmer during training and testing procedures. Things will change if the state feed to the agent is the raw observation of the screenshot we can see; distance between the position of the car and the target flag can be extracted as the feature of the current state.

Other exploration algorithms, to a certain degree, can jump out of the trap. For endogenous exploration such as count-based methods, evolutionary computation techniques, and hindsight experience replay, taking the states of the whole trajectory/episode into consideration may be efficient. Exogenous exploration, which has no relationship to the inner model of the environment, may not face this dilemma.

Exogenous exploration suffers from more outlier effectiveness such as action perturbation [2, 3, 15, 16], Bayesian uncertainty estimation [17–20], parameter space noise [21], or specified reward [22].

Action perturbation exploration [23], alias of sophisticated/dithering exploration strategies, executes exploration process relying on dithering strategy, such as a random selection of the valid actions decided by a probability *ϵ* at the current step in the case of DQN [2, 3]. In the case of deep deterministic policy gradient (DDPG) [15, 16], the agent executes exploration by adding limited noise (maybe Gaussian noise or the more advanced Ornstein–Uhlenbeck noise) to action, which leads to an optimal state-action value at certain step. These strategies suffer inefficient performance in the case of RL problems with multidimensional continuous actions. Gaussian noises or OU noise may be suboptimal, and in practice, however, the hyperparameters which greatly affect the results are difficult to tune. Bayesian uncertainty estimation [17–20] utilized the bootstrap with random initialization, evaluated the uncertainty of neural networks with low computational cost, and made further improvement on deep exploration.

Exogenous exploration strategies act more universally, as they do not rely on the properties of the environments, while the endogenous exploration strategies need more specific design to adapt the environment to be confronted.

In this paper, we introduce a more general frame to make the best of both endogenous exploration and exogenous exploration, which encourage the agent to explore efficiently through the intrinsic reward signal produced by states and encourage the reward signal coming from the diverse goal imagination inspired by the goal exploration processes [23, 24] to interact with a trap group that may be encountered in environment.

## 2. Related Work

Evolutionary computation techniques, focusing on the exploration phase that can be archived to episode-based intrinsic exploration, have emerged as a convincing competitor of deep RL in the continuous action domain [23, 25–28].

Due to more attention to exploration, evolutionary computation techniques search policy directly in the policy parameter space, which results in a good performance in hard exploration situations such as rare reward environment or deceptive reward environment. Compare to SGD-based methods, the evolutionary computation techniques are generally less sample efficient as they lack gradient computations.

Pseudocount-based method, drawing inspiration from the intrinsic motivation literature, combined a mixed Monte Carlo update with a generated exploration bonus to achieve state-of-the-art on the notorious Montezuma's Revenge at that time [4]. The critical pseudocount was derived from an arbitrary density model, which is a generated model to measure the uncertainty of the input state and is utilized by the pleasant theoretical guarantees of count-based exploration methods. Proof was given to demonstrate the close relationship between pseudocounts and information gain, which is widely applied to calculate novelty or curiosity. By introducing an information/prediction gain to measure the log-probability's delta value of two assignments, the authors consequently set information/prediction gain as intrinsic reward to perform count-based exploration.

Exploration with Exemplar (EX2) Models algorithm assessed how simple it is to discriminate between current state and states seen previously and evaluated states' novelty by the simplicity [29].

Reference [6] applied the misprediction error of a learned representation of states to estimate states' novelty. The agent was given exploration bonuses for visiting novel states. In this setting, the agent trained a dynamics model through the learned representation.

## 3. Preliminaries

Consider a Markov decision process (MDP), defined by the tuple (*S*, *A*, *T*, *R*, *γ*). *S* represents state spaces; A represents action spaces. *T* : *S* × *A* × *S*⟶[0; 1] represents the transition distribution which is unknown in the reinforcement learning setting; reward function *R* : *S* × *A* × *S*⟶*ℝ* is unknown, and the value at each time step can be queried through the agent-environment interaction; *γ* is the discount factor to control the importance of future versus immediate rewards.

In reinforcement learning, the agent learns to maximize the expected sum of discounted rewards, *π*^*∗*^=argmax_*π*_*𝔼*_*τ*∼*π*_[∑_*t*=0_^*T*^*γ*^*t*^*R*(*s*_*t*_, *a*_*t*_)], where *τ* denotes a trajectory (*s*_0_, *a*_0_,…, *s*_*T*_, *a*_*T*_) and *π*^*∗*^ is the optimal policy.

Deep deterministic policy gradient (DDPG) is policy-based reinforcement learning. Unlike the value-based DQN agent which chooses action relying on value estimation, the DDPG agent's action is directly computed by a policy *π*, mapping states to a probability distribution over the actions *π* : *S*⟶*P*(*A*). The action-value function *Q*^*π*^(*s*_*t*_, *a*_*t*_)=*𝔼*_*π*_[*R*_*t*_*|s*_*t*_, *a*_*t*_] depicts the expected return of (*s*_*t*_,  *a*_*t*_) under policy *π*. The DDPG agent consists of an actor function *μ*(*s|θ*^*μ*^) (acting as a policy) and a critic function *Q*(*s*,  *a*) (acting as a value estimator). Parameterized actor function *μ*(*s|θ*^*μ*^) maps states to a specific action under the current parameterized policy and makes updates according to the chain rule with respect to the actor parameters.

(1) $$\begin{array}{c} \nabla \mu ={𝔼}_{\mu {}^{\prime }}{\left[\nabla_{a}Q\left(s,a|\theta^{Q}\right)\right)|}_{s=st,a=\mu \left(st\right)}\nabla \theta_{\mu }\mu {\left(s|\theta^{\mu }\right)|}_{s=st}. \end{array}$$

The critic function *Q*(*s*,  *a*) is updated according to Bellman equation as in deep Q-learning. Unlike widely used *ϵ*-greedy strategy, in this work exploration policy is defined as *μ*′(*s*_*t*_)=*μ*(*s*_*t*_*|θ*)+*N*, adding noise sampled from a noise process *N* to the actor policy.

## 4. Count-Based Exploration and Episodic Memory

In low-dimensional Markov decision processes, table reinforcement learning incorporated within count-based exploration works well for states of the Markov decision processes [30] that can be easily exhausted. It is generally accepted that count-based exploration strategies turn inefficient when applied to high-dimensional Markov decision processes (generally high-dimensional state spaces, continuous action spaces, or both) since most states occur only once in deep reinforcement learning. Exploration methods widely applied in deep reinforcement learning rely on heuristic intrinsic motivation to explore unseen states or unreached parts of one state [30].

It is verified that the hippocampus together with the related internal temporal lobe structure in brain supports fast learning. The laboratory rat may be lost in navigation task due to its lesioned hippocampus or temporal lobe. Learning mechanism of the hippocampus is generally recognized as instance-based, while the cortex learns to generalize the representation of input distribution relatively.

The episodic memory module simulates the work of the hippocampus in the human brain. This is exactly the memory of past experience. It seems naturally and logically to apply episodic memory to count the situations encountered. Therefore, we use the contextual memory module to remember the states that the agent has encountered, as a count of states, and the purpose of exploration is to reduce the probability of encountering these states again. The purpose of exploration is to counter the episodic memory.

Inspired by model-free episodic control [31], we set the reward of the last state of one rollout as 1, *R*_*c*_(*T*) = 1; when discount factor *γ*=1, state value of each state experienced in the rollout can be *C*(*s*_*i*_)=1,  *i*=1...*T*; in other words, the count value of each state is 1, *C*_count_(*s*_*i*_)=1. The C value is updated as follows:

(2) $$\begin{array}{c} C_{\text{count}}\left(s_{t},\;a_{t}\right)\leftarrow \left\{\begin{array}{cc} R_{ct}, & \text{if}\left(s_{t},\;a_{t}\right)\notin C_{\text{count}},\\ \max\left\{C_{count}\left(s_{t},a_{t}\right),R_{ct}\right\}, & \text{otherwise.} \end{array}\right) \end{array}$$

When encountering a state that has never been seen before, the *C*_*t*_ value is assigned to *R*_*c*_(*t*).

(3) $$\begin{array}{c} C_{\text{count}}\left(s,\;a\right)\;=\left\{\begin{array}{cc} \frac{1}{k}\sum_{i=1}^{k}C_{\text{count}}\left(s^{\left(i\right)},\;a\right), & \text{if}\left(s,\;a\right)\notin C_{\text{count}}\text{,}\\ C_{count}\left(s,\;a\right), & \text{otherwise.} \end{array}\right) \end{array}$$

A critical process is to make decisions on when to explore and when to exploit; an indicator is designed to measure the exploration degree of current state, which is set to the ratio of delta between the maximum and the minimum counter; the agent explores when indicator is greater than the previously set threshold value; otherwise it exploits.

(4) $$\begin{array}{c} \frac{\max C_{count}\left(s_{t}\right)-\min C_{count}\left(s_{t}\right)}{\max C_{count}\left(s_{t}\right)}\leq \zeta . \end{array}$$

We attach state counter to episodic memory, benefiting from the mechanism of episodic control algorithm. During the process of searching and updating, there is no need to establish another tree structure or to occupy other extra computing resources or memory.

## 5. Experiments

To verify in practice whether CounterEM learns more data efficiently, Atari Learning Environment [32, 33] which consists of various reward structures and exploration levels was chosen as a problem domain. We test our approach on Atari games that contain a series of interesting tasks such as sparse rewards and scores across different games. Pervious work had done a lot to apply the commonly used algorithms such as DQN and A3C and their variants in Atari Learning Environment and can be taken as baselines.

Reference [34] reproduces taxonomy of games in Atari Learning Environment on the basis of their exploration difficulty. Rough taxonomy of the games of Atari is “sparse” or “dense” rewards which depict the game's reward structure qualitatively. Limited by computing resources, we chose the seven notorious “sparse” rewards hard exploration games: Freeway, Gravitar, Montezuma's Revenge, Pitfall!, Private Eye, Solaris, and Venture; ten “dense” rewards hard exploration games: Alien, Amidar, Bank Heist, Frostbite, HERO, Ms. Pac-Man, Q*∗*bert, Surround, Wizard of Wor, and Zaxxon; and ten easy exploration games: Bowling, Breakout, Pong, Space Invaders, Boxing, Seaquest, Skiing, Demon Attack, Enduro, Gopher.

### 5.1. Experimental Parameters

For A3C, we run 100 rollout steps before being trained with 50 random batches of samples from the replay buffer. The cycle is repeated 20 times (2000 steps in the environment) before A3C is evaluated offline on 10000 steps (10 episodes). Replay buffer is a sliding window of size 10^6^.

20 different seeds were used to reduce the variance of statistically different results. The inverse model first maps the input state (*s*_*t*_) to a feature vector *ϕ*(*s*_*t*_) using a series of two hidden layers of size (128, 128). For the inverse model, *ϕ*(*s*_*t*_) and *ϕ*(*s*_*t*+1_) are concatenated into a single feature vector and passed as inputs into a fully connected layer of 64 units. The forward model is constructed by concatenating Φ(*st*) with *at* and passing them into a sequence of two fully connected layers with 64 and 128 units, respectively. The value of *β* is set to 0.2, while *λ* is set to 0.1. The batch size is set to 64, the discount factor is set to 0.99, and the actor and critic networks are designed with the same structure of two hidden layers of size (64, 64) with RELU activation functions. What is different is their output layer activation function; actor network output layer activation function is tanh while the critic network is linear.

The learning rates are 10−4 and 10−3, respectively, and Adam is used to optimize the loss function. The OU noise used in the A3C and the variant DQN algorithms linearly decreased from 0.9 at the first step to 0.1 at the final step. The performance was reported over 100 evaluation episodes of the best policy found during training process; each episode is set to 500 steps on the games.

### 5.2. Results

Table 1 summarizes the experimental results and data efficiency. CounterEM (NEC) and CounterEM (MFEC) significantly outperformed all other algorithms at small training step (less than 10 million frames). The gap is especially observed before 20 million frames (Algorithms 1 and 2).

Equipped with CounterEM, MFEC and NEC have a clear advantage in the initial learning stage, especially before 4 million frames. With the increase of training frames, CounterEM's efficiency gradually decreases. However, it is worth noting that CounterEM (NEC) outperformed the other baseline algorithms, training 40 million frames at its 10 million frames, which means more than 100 hours of training time.

In most of the Atari games, CounterEM (NEC) outperformed CounterEM (MFEC) on average, and both learned significantly faster in the initial phase than other baseline algorithms (see Table 2). At 2 million frames, CounterEM (MFEC) outperformed NEC. MFEC and NEC without CounterEM applied inefficient random exploration, which becomes even less efficient as the number of actions increases. Thanks to proven count-based exploration methods, CounterEM directs agents to explore unseen or rare-seen states to obtain high rewards quickly. However, when the training step increases up to a certain threshold, which may be positively correlated to the dimensions of states and actions, the superiority of CounterEM may weaken.

It is worth noting that, in order to ensure the stability of training, the baseline algorithms A3C and DQN and related variant algorithms need to crop the reward to the range of [−1, 1] [2, 3]. NEC and MFEC do not need reward clips, and therefore CounterEM (NEC) and CounterEM (MFEC) do not require reward clips. This resulted in quality changes in behavior and better performance than other games that required editing (such as Alien, Frostbite, Pac-Man, Bowling, and HERO). The counter estimator is naturally set to the [−1, 1] range, but this does not affect the agent's learning efficiency in these games because we do not use the counter estimator directly in the *Q* calculation.

### 5.3. Experiment for Object Detection

To test our module in high dimensions, we turn to object localization/object detection which plays an important role in the computer vision field. RL-based target detection and target tracking usually use the standard A3C algorithm, and they pay more attention to the design of the framework and network structure, while action disturbance is used for exploration. As a very important link in RL, exploration also plays an important role in this application field. Its goal is to place bounding boxes in a given image around the instances of predefined object class, such as faces, ships, and desktops. During localization process, detectors analyze the scanning windows of the input image, while the transformation of windows is guided by scales and locations. Most state-of-the-art solutions for object detection are bottom-up region proposals [35, 36]; thousands of windows were selected and evaluated one by one. These bottom-up methods were accelerated by the advancement of convolutional neural networks (CNNs) and parallel computing benefits from rapid expansion of graphic processing unit (GPU) [37–40].

Current active search methods, reformulated for learning a navigation strategy, based on the DQN frame, artificially designed several actions (horizontal/vertical moves in fixed pixels, scale changes in fixed scale related to the pixels, aspect ratio changes in fixed ratio related to the pixels, trigger) to form an action set [41–47]. Agent selected action (*a*) that generates the max estimated action value (*Q*); that is to say, the policy *π* = *P*(*a|s*) would not exist independently of the action-value estimation, which leadd to continuous action space situation beyond the off-policy algorithm as maximum action value is not easy to figure out.

#### 5.3.1. State

The state of the MDP consists of the whole image feature vector, current time step window feature vector, and history of performed actions in current episode. These three elements are simply concatenated into a new vector to represent the state. The features are extracted using a pretrained VGG-16 model [48] for both the whole image and current window. Feature vector of layer fc6 *r*_*t*_+1 was applied in our experiments, and the VGG-16 was pretrained on ImageNet.

#### 5.3.2. Action

An action space *A*(*s*) defines the legal action in any given state *s* ∈ *S*; at each time step, the agent performs action to deploy the box which surrounds the object. In the 2D object detection application, four possible actions, up, down, left, and right, allow for pixel-wise movement being universal solution.

#### 5.3.3. Reward Function

The agent receives a new visual observation of the environment *s*_*t*+1_ and a reward signal *r*_*t*+1_ when performing the action obtained from the agent.

The agent makes decision to maximize the sum of the reward signal *R*=∑_*i*_*r*_*i*_, while in application fields, it is usually very sparse and hysteric.

To simulate the common situation, in our object detection experiment, we set *r*_*T*_=1 only when object is classified correctly and 0 otherwise.

#### 5.3.4. Results

Figure 1 is an experimental comparison diagram of several applications in the CV field. We use the three different exploration methods of OU noise [15, 16], GEP [23], and Reachable [34, 49–53] for comparison with our CounterEM method, in pedestrian tracking and face detection. Experiments show that CounterEM can get good rewards quickly.

## 6. Conclusions

Episodic memory can be used for episodic control and can achieve good results in some RL application situations. In the case of relatively easy exploration or nonsparse reward, the agent can find the path of high reward very smoothly, even when reward is sparse. The problems of reward and hard exploration are dependent more on the strategy of exploration. In this article, we modified the episodic memory module to pseudocount state, so as to realize a pseudocount-based exploration strategy. The experiment shows that our algorithm can achieve good results in OpenAI games as well as computer vision applications such as object detection and object tracking. In the next step, we plan to expand the counter episodic memory to continuous episodic control. Dual networks seem to be a feasible solution, because their inputs are all the states at certain time, and their embeddings are consistent.

## Figures and Tables

**Figure 1:** Sum reward in computer vision applications.

**Algorithm 1:** Exploration for countering model-free episodic control.

**Algorithm 2:** Exploration for countering neural episodic control.

**Table 1:** Median across games of human-normalized scores for listed algorithms at different training frames.

Frames (M)	Nature DQN (%)	Retrace(*λ*) (%)	A3C (%)	MFEC (%)	CounterEM (MFEC) (%)	NEC (%)	CounterEM (NEC) (%)
1	−0.7	−0.4	0.4	12.8	20.1	16.7	29.6
2	0.0	0.2	0.9	16.7	29.1	27.8	37.6
4	2.4	3.3	1.9	26.6	36.2	36.0	48.4
10	15.7	17.3	3.6	45.4	52.5	54.6	69.3
20	26.8	30.4	7.9	55.9	66.1	72.0	77.6
40	36.7	60.5	18.4	61.9	70.0	83.3	84.5

**Table 2:** Mean human-normalized scores for listed algorithms at different training frames.

Frames (M)	Nature DQN (%)	Retrace(*λ*) (%)	A3C (%)	MFEC (%)	CounterEM (MFEC) (%)	NEC (%)	CounterEM (NEC) (%)
1	−10.5	−10.5	5.2	28.4	40.8	45.6	61.7
2	−5.8	−5.4	8.0	39.4	68.3	58.3	84.9
4	8.8	6.2	11.8	53.4	88.4	73.3	97.3
10	51.3	52.7	22.3	85.0	100.1	99.8	115.4
20	94.5	237.7	59.7	113.6	117.9	121.5	122.8
40	151.2	386.5	255.4	142.2	148.1	144.8	150.0

## Data Availability

The game data used to support the findings of this study are included within the article.
